# Correlation between Coagulation Fibrinolysis Function and Outcomes during Hospitalization in Patients with Severe Traumatic Hemorrhagic Shock

This article has been retracted.

**DOI:** 10.1155/2022/3775868

**Published:** 2022-06-30

**Authors:** Louwei Zhang, Maosheng Lin, Xuhua Tang, Yejiang Tang

**Affiliations:** Department of Emergency Medicine, Zhuji Affiliated Hospital of Shaoxing University, Zhuji 311800, Zhejiang, China

## Abstract

**Objective:**

To analyze the correlation between coagulation fibrinolysis function and outcomes during hospitalization in patients with severe traumatic hemorrhagic shock.

**Methods:**

A retrospective collection was performed on the clinical data of 106 patients with severe traumatic shock admitted to the hospital between January 2020 and January 2022. According to the injury severity score (ISS), they were divided into the S1 group (ISS <25 points, *n* = 70) and the S2 group (ISS ≥25 points, *n* = 36). The prothrombin time (PT), fibrinogen (Fib), thrombin time (TT), and activated partial thromboplastin time (APTT) were detected by the coagulation assay. The aD-dimer (D-D) was detected by an enzyme-linked immunosorbent assay. Antithrombin activity (AT : A) and plasminogen activity (PLG : A) were detected by the chromogenic substrate method. The relationship between coagulation fibrinolysis indexes and injury severity was analyzed by Spearman's correlation analysis. The predictive value of coagulation fibrinolysis indexes for outcomes of patients with severe traumatic hemorrhagic shock was evaluated by receiver operating characteristic (ROC) curves.

**Results:**

The levels of PT, APTT, D-D, TT, AT : A and PLG : A in the S2 group were higher than those in S1 group, while the Fib level was lower than that in the S1 group (*P* < 0.05). A Spearman's analysis showed that PT, APTT, TT, D-D, AT : A, and PLG : A were positively correlated with injury severity (*P* < 0.05), while Fib was negatively correlated with it (*P* < 0.05). Among the 106 patients, there were 89 survived cases and 17 died cases. The levels of PT, APTT, D-D, AT : A and PLG : A in the death group were lower than those in the survival group, while the Fib level was higher than that in the survival group. The results of ROC curve analysis showed that serum PT, APTT, Fib, TT and D-D were of predictive value for outcomes (*AUC* = 0.713, *AUC* = 0.683, *AUC* = 0.712, *AUC* = 0.761, *AUC* = 0.730, *AUC* = 0.765, *AUC* = 0.673, *P* < 0.05), and cutoff values were 20.29 s, 34.79 s, 3.54 g/L, 20.97 s, 1.42 *μ*g/L, 73.53% and 63.97%, respectively.

**Conclusion:**

There is coagulation and fibrinolysis dysfunction in patients with severe traumatic hemorrhagic shock, which is related to injury severity. The coagulation fibrinolysis indexes have a certain predictive value for outcomes of patients.

## 1. Introduction

Traumatic shock is a combination of factors such as severe violent blows on the body, major organ damage, and massive hemorrhage. The body's decompensation syndrome is formed.. Therefore, the etiology and pathology of traumatic shock are more complicated than simple hemorrhagic shock. Severe traumatic hemorrhagic shock occurs when the patient bleeds a lot, blood volume decreases, and local tissue necrosis occurs due to severe impact by external force in a short time [1]. The main clinical presentations are severe pain, shortness of breath, pale face, weakened jugular vein pulse, and confusion. Due to insufficient systemic tissue perfusion, metabolic disorders, impaired cell ischemia, hypoxia, and severe traumatic hemorrhagic shock, it is prone to cause damage to multiple organs [2, 3]. The condition of patients is complex and in danger, with many early complications and high mortality, which makes it a severe illness in the hospital. Effective treatment should be given to reduce the complications and improve the patient's prognosis. The pathophysiological process of traumatic ischemic shock is complex, and the coagulation chain reaction that can be triggered by shock plays an important role in the disease [4]. Results of some studies have shown [5] that when the patient suffers severe liver damage, the incidence of consumptive coagulopathy will reach as high as 50%. However, the impact of the shock on the coagulation and fibrinolysis systems of patients with traumatic blood loss and the relationship between shock and patient outcomes remains controversial [6, 7]. The bodies of patients with shock are in a hypercoagulable state and are prone to suffering thrombosis as the high-intensity injury damages the repair function of the body seriously and the coagulation and fibrinolysis function are gradually disturbed [8]. If severe traumatic hemorrhagic shock onsets rapidly and the treatment is not timely, the risk of death will be greatly increased. This study analyzed the changes in coagulation and fibrinolysis in patients with severe traumatic shock and the association between the changes and the outcome in order to provide guidance for the clinical.

## 2. Clinical Data and Methods

### 2.1. General Information

The clinical data of 106 patients with severe trauma shock admitted to our hospital from January 2020 to January 2022 were retrospectively selected. Patients were divided into S1 group (ISS score <25, *n* = 70) and S2 group (ISS score ≥25, *n* = 36) based on the severity of trauma (ISS). Group S1 had 38 males and 32 females, aged 12–70 years, with an average age of 49.64 ± 9.78 years. Causes of trauma were traffic accident injury in 15 cases, fall injury in 22 cases, traffic accident injury in 16 cases, and knife stabbing injury in 17 cases; trauma site: brain injury in 12 cases, chest injury in 23 cases, and abdominal injury was the main injury in 17 cases and 18 cases were mainly spinal and limb injuries. In the S2 group, there were 20 males and 16 females, aged 15–70 years, with an average age of 51.21 ± 9.36 years. Causes of trauma: 9 cases of traffic accidents, 12 cases of falling from height, 7 cases of traffic accidents, and 8 cases of knife stabbing; trauma site: brain injury in 5 cases, chest injury in 14 cases, and abdominal injury in 14 cases out of which 9 cases were mainly sprains and 8 cases were mainly spinal and limb injuries. Inclusion criteria were meeting the diagnostic criteria for severe traumatic hemorrhagic shock [9]; ISS score ≥16 points on admission; survival time after rescue ≥24 hours. Exclusion criteria were patients with liver and kidney dysfunction; patients with mental disorders; and patients with missing clinical data. There was no significant difference in age, gender, trauma cause, and trauma site between the S1 and S2 groups (*P* > 0.05). This study has been approved by the Medical Ethics Committee of our hospital.

### 2.2. Detection of Serum Coagulation and Fibrinolysis Indexes

The next day, after the patients were enrolled, 5 mL of peripheral venous blood was collected in the fasting state, and the supernatant was collected after centrifugation (1200 g, 8 cm, 5 min). Prothrombin time (PT), fibrinogen (Fib), thrombin time (TT), and activated partial thromboplastin time (APTT) were detected by coagulation method. D-dimer (D-dimer, D-D) was detected by an enzyme-linked immunofluorescence assay. The instruments and related kits were purchased from Beijing Boaosen Biotechnology Co., Ltd. The antithrombin activity (AT : A) and plasminogen activity (PLG : A) were detected by the chromogenic substrate method. The kits were purchased from Wuhan Purity Biotechnology Co., Ltd., and the operations were carried out in strict accordance with the kit instructions.

### 2.3. Statistical Processing

The SPSS 22.0 software was used for statistical analysis. All experimental data conformed to normal distribution, and measurement data were presented as mean ± standard deviation ($\bar{X}\pm S$), and the two-sample independent *t*-test was used to compare the differences between groups. The enumeration data were expressed as [cases (%)], and the difference between the two groups was compared by the *χ*2 test. Spearman's correlation was used to analyze the relationship between the coagulation and fibrinolysis indexes and the severity of the injury. The receiver operator characteristic curve (ROC) was used to measure the predictive effect of coagulation and fibrinolysis indexes in patients with severe traumatic hemorrhagic shock. The test level was *α* = 0.05, and *P* < 0.05 indicated that the data had a significant statistical difference.

## 3. Result

### 3.1. Comparison of Serum Coagulation and Fibrinolysis Indexes in Each Group

The levels of PT, APTT, D-D, TT, AT : A, and PLG : A in group S2 were higher than those in group S1, the level of Fib was lower than that in group S1, and the difference was statistically significant (*P* < 0.05), as shown in Table 1 and Figure 1.

### 3.2. Correlation Analysis between the Severity of Injury and Coagulation and Fibrinolysis Indexes in Patients

The result of Spearman analysis showed that PT, APTT, TT, D-D, AT : A, and PLG : A were positively correlated with injury severity (*P* < 0.05), and Fib was negatively correlated with injury severity (*P* < 0.05). As shown in Table 2 and Figure 2.

### 3.3. Comparison of Serum Coagulation and Fibrinolysis Indexes between Death Group and Survival Group

The patient's survival time within three months was recorded. Among the 106 patients, 89 survived and 17 died. The levels of PT, APTT, D-D, AT : A, and PLG : A in the death group were lower than those in the survival group, and the Fib level was higher than that in the survival group (*P* < 0.05). As shown in Table 3.

### 3.4. Predictive Value of Coagulation and Fibrinolysis Indexes on Patient Outcome

The ROC results show that serum PT, APTT, Fib, TT, D-D, AT : A and PLG : A could all predict the outcome of patients (AUC = 0.713, AUC = 0.683, AUC = 0.712, AUC = 0.761, AUC = 0.730, AUC = 0.765, AUC = 0.673, *P* < 0.05), At this time, the cutoff values were 20.29 s, 34.79 s, 3.54 g/L, 20.97 s, 1.42 *μ*g/L, 73.53%, and 63.97%, respectively, as shown in Figure 3 and Table 4.

## 4. Discussion

The main pathophysiological change of traumatic hemorrhagic shock is the mismatch between blood volume and vascular volume, resulting in insufficient perfusion of peripheral tissues and inducing changes in microcirculation, abnormal oxygen metabolism, inflammatory response, coagulation disorders, and secondary damage to organs [10, 11]. The disease has the characteristics of a short-term onset and high mortality. Therefore, clinicians should take timely intervention measures to save the patient's life as much as possible.

The coagulation and fibrinolysis systems are in a state of dynamic equilibrium under physiological conditions. When the body is injured, the balance system is disrupted, and the coagulation and fibrinolysis systems are activated [12]. In this study, the levels of PT, APTT, D-D, TT, AT: A, and PLG: A in group S2 were higher than those in group S1, and the level of Fib was lower than that in group S1. D-D is a specific product after the degradation of cross-linked fibrin, which mainly reflects the function of fibrinolysis. The increase in its concentration indicates that the fibrinolytic system and the coagulation system are activated [13]. Fib is a protein with a coagulation function that is synthesized by the liver [14]. PT mainly reflects whether the extrinsic coagulation is normal or not and reflects the content of plasma factors II, V, VII, and X, and its prolongation is seen in congenital coagulation factor deficiency [15]. TT refers to the blood coagulation time after adding standardized prothrombin to plasma, which reflects the anticoagulant substances in the body, and its prolongation indicates hyperfibrinolysis [5]. During traumatic hemorrhagic shock, the coagulation and fibrinolysis systems, as the main systems involved in stress and hemostasis, are activated urgently and play an important role in the occurrence and development of shock. Its changes within a certain range have a positive effect on hemostasis and antishock [16]. However, if the factors that induce the coagulation and fibrinolysis system are excessive or continuously stimulated, it may increase the degree of shock. This study shows that the balance of coagulation and fibrinolysis in patients with traumatic hemorrhagic modification is disrupted, and the dysfunction of coagulation and fibrinolysis becomes more serious with the aggravation of the disease. The results of Spearman's correlation analysis showed that PT, APTT, TT, D-D, AT: A, and PLG: A were positively correlated with injury severity, and Fib was negatively correlated with injury severity. Previous studies have shown [17] that the more severe the injury is in patients with traumatic hemorrhage, the more likely they are to have coagulation and fibrinolysis dysfunction, which coincides with the results of this study. The results indicate that the coagulation system is continuously activated in the acute stage of severe trauma, the patient's blood is in a state of hypercoagulation and high viscosity, and the risk of intravascular coagulation and thrombosis is greatly increased. Therefore, at this time, the blood volume of the patient should be replenished in a timely and effective manner, which can help the patient return to a normal physiological state and gradually seek medical treatment for the pathological process. At the same time, during the treatment process, attention should be paid to the coagulation and fibrinolysis function status of patients, and interventions such as early coagulation substrates should be given. At the same time, this study also found that among the 106 patients, 89 survived and 17 died. The levels of PT, APTT, D-D, AT : A, and PLG : A in the death group were lower than those in the survival group, and the Fib level was higher than that in the survival group, indicating that the coagulation and fibrinolysis indexes of the patients in the death group were significantly abnormal. Analysis of ROC results showed that serum PT, APTT, D-D, AT : A, and PLG : A all had a certain value in predicting patient outcomes. Previous studies have shown [18] that the abnormality of coagulation and fibrinolysis in patients with traumatic brain injury in the early post-injury period is related to the severity of the traumatic brain injury and has a certain evaluation value for the patient's condition and prognosis, which is basically consistent with this study. Therefore, coagulation and fibrinolysis dysfunction after traumatic blood loss is an important reason for the aggravation and death of shock patients. Paying attention to the changes in coagulation and fibrinolysis indexes in shock patients caused by traumatic blood loss and early intervention are of great significance in reducing the mortality of patients.

In conclusion, the blood of patients with severe traumatic hemorrhagic shock is in a hypercoagulable state, with continuous activation of the coagulation system and hyperfibrinolysis, increasing the risk of secondary thrombosis and bleeding, and the patient's state increases with the severity of the injury. Coagulation and fibrinolysis indexes are of great significance for assessing the severity of injury and predicting the prognosis of patients. This study has a certain guiding significance for clinical treatment of patients with severe traumatic shock and improvement of prognosis, but there are still shortcomings: the research is still in the preliminary stage, and the specific mechanism of action on the coagulation and fibrinolysis system after traumatic blood loss has not been deeply analyzed. Due to the small number of research samples, there may be errors in the analysis results, and a large number of subsequent clinical data are required for verification.

## Figures and Tables

**Figure 1:** Comparison of serum coagulation and fibrinolysis indexes in each group. PT: prothrombin time, APTT: activated partial thromboplastin time, Fib: fibrinogen, TT: thrombin time, D-dimer, D-D: D-dimer, AT: A: antithrombin activity, and PLG : A: plasminogen activity; ^*∗*^*P* < 0.05 compared with the S1 group.

**Figure 2:** Comparison of serum coagulation and fibrinolysis indexes in each group. PT: prothrombin time, APTT: activated partial thromboplastin time, Fib: fibrinogen, TT: thrombin time, D-dimer, D-D: D-dimer, AT: A: antithrombin activity, and PLG : A: plasminogen activity; ^*∗*^*P* < 0.05 compared with the survival group.

**Figure 3:** Predictive effect of coagulation and fibrinolysis indexes on patient outcomes.

**Table 1:** Comparison of serum coagulation and fibrinolysis indexes in each group ($\bar{X}\pm S$).

Group	Number of cases	PT (s)	APTT (s)	Fib (g/L)	TT (s)	D-D (mg/L)	AT : A (%)	PLG : A (%)
Group S1	70	17.54 ± 1.82	29.81 ± 3.04	4.41 ± 0.57	17.25 ± 1.87	1.03 ± 0.12	76.13 ± 7.74	77.33 ± 7.82
Group S2	36	21.46 ± 2.33	35.72 ± 3.61	3.28 ± 0.39	23.86 ± 2.46	1.44 ± 0.15	72.58 ± 7.36	61.85 ± 6.32
*t* value		9.527	8.886	10.668	15.441	15.276	2.273	10.270
*P* value		<0.001	<0.001	<0.001	<0.001	<0.001	0.025	<0.001

**Table 2:** Correlation analysis between the severity of injury and coagulation and fibrinolysis indexes in patients.

Indicator	Severity of trauma	
	*r*	*P*
PT	0.542	0.036
APTT	0.611	0.027
TT	0.654	0.041
Fib	−0.586	0.003
D-D	0.637	0.017
AT : A	0.589	0.042
PLG : A	0.609	0.038

**Table 3:** Serum coagulation and fibrinolysis indexes of death group and survival group ($\bar{X}\pm S$).

Group	Number of cases	PT (s)	APTT (s)	Fib (g/L)	TT (s)	D- (*μ*g/L)	AT : A (%)	PLG : A (%)
Survival group	89	18.06 ± 1.96	30.86 ± 3.12	4.59 ± 0.51	18.63 ± 2.03	1.08 ± 0.12	75.89 ± 7.62	74.58 ± 7.68
Death group	17	22.85 ± 2.35	36.87 ± 3.74	3.20 ± 0.34	24.18 ± 2.62	1.59 ± 0.16	69.84 ± 7.14	58.64 ± 6.23
*t* value		8.927	7.045	10.767	9.837	15.174	3.028	8.056
*P* value		<0.001	<0.001	<0.001	<0.001	<0.001	0.003	<0.001

**Table 4:** Predictive effect of coagulation and fibrinolysis indexes on patient outcome.

Indicator	AUC	Standard error	Sensitivity (%)	Specificity (%)	Cutoff value	95%CI	*P*
PT	0.713	0.094	70.59	79.78	20.29 (s)	0.617∼0.797	<0.05
APTT	0.683	0.081	64.71	80.90	34.79 (s)	0.586∼0.700	<0.05
Fib	0.712	0.088	76.47	78.65	3.54 (g/L)	0.616∼0.796	<0.05
TT	0.761	0.069	76.47	69.66	20.97 (s)	0.669∼0.839	<0.05
D-D	0.730	0.080	70.59	84.27	1.42 (*μ*g/L)	0.635∼0.811	<0.05
AT : A	0.765	0.074	76.47	75.28	73.53 (%)	0.672∼0.842	<0.05
PLG : A	0.673	0.072	70.59	65.17	63.97 (%)	0.575∼0.761	<0.05

## Data Availability

The data can be obtained from the author upon reasonable request.
